The article "A Study on the Preventive Effect of Esketamine on Postpartum Depression (PPD) after Cesarean Section" was retracted in 2023. Reasons: unreliable results or conclusions; concerns about the data; concerns about the peer review; concerns about the citations.

# A Study on the Preventive Effect of Esketamine on Postpartum Depression (PPD) after Cesarean Section

**DOI:** 10.1155/2022/1524198

**Published:** 2022-08-08

**Authors:** Qiwei Wang, Maoxin Xiao, Hao Sun, Pengcheng Zhang

**Affiliations:** ^1^Department of Anesthesiology, The Fourth Hospital of Shijiazhuang, Shijiazhuang, 050000 Hebei, China; ^2^Department of Anesthesiology, The Eighth Hospital of Shijiazhuang, Shijiazhuang, 050000 Hebei, China

## Abstract

**Objective:**

The purpose of this study is to explore and analyze the preventive effect of esketamine on postpartum depression (PPD) after cesarean section.

**Methods:**

A total of 138 puerperae who underwent cesarean section in our hospital from February 2020 to January 2022 were selected as the research subjects. The control group was given intravenous injection of 2 ml of normal saline after the fetus was delivered. Meanwhile, the observation group was given intravenous injection of a small dose of esketamine (esketamine 0.5 mg/kg+ 2 ml of normal saline) after the delivery of the fetus. The changes of blood pressure and heart rate, the Edinburgh Postnatal Depression Scale (EPDS) questionnaire scores and the incidence of postpartum depression were compared between the two groups. At the same time, the incidence of postoperative adverse events in the two groups was observed.

**Results:**

There was no significant difference in systolic blood pressure (SBP), diastolic blood pressure (DBP), and heart rate (HR) between the two groups at T1-T3 (*P* > 0.05). Compared with the control group, the SBP, DBP, and HR at T4 and T5 in the observation group were higher (*P* < 0.05). There was no significant difference in SBP, DBP, and HR at T3, T4, and T5 in the observation group (*P* > 0.05). Compared with T3, SBP, DBP, and HR were lower in control group T4 and T5, respectively. There was no significant difference in the EPDS scores between the two groups on the 1st day before delivery (*P* > 0.05). The EPDS scores of the two groups were higher at 3d postpartum and 42d postpartum, respectively, than at 1d before delivery. The EPDS scores of the observation group at 3d and 42d after delivery were lower than those in the control group (*P* < 0.05). Compared with the control group, the incidence of postpartum depression was higher in the observation group at 3 days postpartum and 1 month postpartum, respectively (*P* < 0.05). There was no significant difference in the incidence of postpartum adverse reactions between the two groups (*P* > 0.05).

**Conclusion:**

The application of esketamine after cesarean section can effectively reduce depression-related scores and the risk of postpartum depression without increasing adverse reactions and has high safety.

The article "A Study on the Preventive Effect of Esketamine on Postpartum Depression (PPD) after Cesarean Section" was retracted in 2023. Reasons: unreliable results or conclusions; concerns about the data; concerns about the peer review; concerns about the citations.

## 1. Introduction

Postpartum depression, also known as postpartum depression, mainly refers to a type of depression that occurs in the puerperium. The main symptoms and manifestations of postpartum depression are different degrees of depression and mental depression. If postpartum depression is not properly dealt with, it will easily lead to the development of the patient's depressive symptoms to a more serious level or even suicide and self-harm, bringing many negative effects and problems to the mother-infant relationship and the infant's emotional and behavioral growth [1]. Therefore, it is of great clinical significance to take active and effective methods to prevent the occurrence of puerperal depression. The traditional antidepressant drugs used in previous clinical work have slow onset of action, poor cure rate, and preventive effect, and it is impossible to judge whether they can be used for safe breastfeeding [2]. In recent years, studies have shown that small doses of esketamine can play a strong analgesic effect. At the same time, the application of esketamine in the treatment of refractory depression and marital form disorder will also play a good role. This study began to apply esketamine after cesarean section to analyze whether it can prevent the occurrence of postpartum depression. The results are reported below.

## 2. Materials and Methods

### 2.1. General Information

A total of 138 puerperae who underwent cesarean section in our hospital from February 2020 to January 2022 were selected as the research subjects. All puerperae were randomly divided into control group and observation group, with 69 cases in each group. The ASA grades of all puerperae were grades I to II, and there was no significant difference in general data between the two groups (*P* > 0.05) (Table 1). Inclusion criteria are as follows: all puerperae who gave birth at term, puerperae who meet the indications for cesarean section, maternal absence of contraindications to spinal canal, and prenatal screening of mothers without severe fetal malformations or defects. Puerperae and their families gave informed consent to this trial. Exclusion criteria are as follows: puerperae with prenatal history of mental illness and brain disease; puerperae who have experienced major life events before birth; maternal coexistence with other types of obstetric diseases, including pregnancy-induced hypertension syndrome, eclampsia, placenta previa, and placental abruption; puerperae with serious comorbidities such as fake Xi'an hyperfunction and high blood pressure were combined; and puerperae with missing clinical data. All the specimens of this study were gotten the informed consent from patients and were approved by the Ethical Committee of Fourth Hospital of Shijiazhuang.

The article "A Study on the Preventive Effect of Esketamine on Postpartum Depression (PPD) after Cesarean Section" was retracted in 2023. Reasons: unreliable results or conclusions; concerns about the data; concerns about the peer review; concerns about the citations.

### 2.2. Methods

All puerperae were given combined spinal-epidural anesthesia treatment, the puerperae were lying on the left side, and puncture treatment was given between the L2-3. After successful epidural puncture, subarachnoid block was administered using the “intra-needle method” with a “pencil tip” spinal needle. After the puncture is successful, turn the bevel of the puncture needle toward the head, and inject 10 mg of bupivacaine (Hunan Kelun Pharmaceutical Co., Ltd., approved by Chinese medicine H43021411) with equal specific gravity at a speed of 10 to 15 s. After injecting the drug, adjust the maternal position to the left lateral decubitus position of 15°, and regulate the anesthesia level at T10. All puerperae selected the same group of obstetricians, made a transverse incision in the pubic bone, and performed cesarean section through the abdominal cavity [3]. The control group was given intravenous injection of 2 ml of normal saline after the fetus was delivered (Beijing Institute of Biological Products Co., Ltd., S10870001). And the observation group was given intravenous injection of a small dose of esketamine after the delivery of the fetus (Esketamine 0.5 mg/kg+ 2 ml of normal saline). No other type of analgesic drugs were used in the two groups of women, and no postoperative analgesia was given.

### 2.3. Observation Indicators

The changes of blood pressure and heart rate, the Edinburgh Postnatal Depression Scale (EPDS) questionnaire scores and the incidence of postpartum depression were compared between the two groups. At the same time, the incidence of postoperative adverse events in the two groups was observed. The perioperative time points were 15 minutes before administration (T1), 5 minutes before administration (T2), during administration (T3), 5 minutes after administration (T4), and 15 minutes after administration (T5). The evaluation indicators of the EPDS questionnaire included 10 items including mood, fun, self-blame, fear, anxiety, insomnia, coping ability, sadness, crying, and suicide. Each item is scored on a 4-point scale, with a score between 0 and 30. The higher the score, the more severe the depressive symptoms. A score of 10 and above is diagnosed as postpartum depression [4]. Common types of adverse reactions include nausea, vomiting, dizziness, and headache.

### 2.4. Statistical Processing

SPSS 23.0 statistical software was used to analyze the data. Three replicates were performed for each experiment. Enumeration data were expressed as %, and *χ*^2^ test was used. Measurement data were expressed as mean ± standard deviation (mean ± sd), *t*-test was used, and *F*-test was used for comparison of multiple groups. Statistical significance was represented by *P* < 0.05.

The article "A Study on the Preventive Effect of Esketamine on Postpartum Depression (PPD) after Cesarean Section" was retracted in 2023. Reasons: unreliable results or conclusions; concerns about the data; concerns about the peer review; concerns about the citations.

## 3. Results

### 3.1. Comparison of Changes in Blood Pressure and Heart Rate between the Two Groups

There was no significant difference in SBP, DBP, and HR between the two groups at T1-T3 (*P* > 0.05). Compared with the control group, the SBP, DBP, and HR at T4 and T5 in the observation group were higher (*P* < 0.05). There was no significant difference in SBP, DBP, and HR at T3, T4, and T5 in the observation group (*P* > 0.05). Compared with T3, the SBP, DBP, and HR were lower in the control group T4 and T5, respectively (*P* > 0.05) (Table 2).

### 3.2. Comparison of EPDS Scores before and after Cesarean Section between the Two Groups

There was no significant difference in the EPDS scores between the two groups on the 1st day before delivery (*P* > 0.05). The EPDS scores of the two groups were higher at 3d and 42d postpartum than those at 1d before delivery. The EPDS score of the observation group was lower at 3d and 42d after delivery than that of the control group at 3d and 42d after delivery, respectively (*P* < 0.05) (Table 3).

### 3.3. Comparison of the Incidence of Depression after Cesarean Section between the Two Groups

The incidence of postpartum depression was higher in the observation group than that in the control group at 3 days postpartum and at 1 month postpartum, respectively (*P* < 0.05) (Table 4).

### 3.4. Comparison of the Incidence of Adverse Reactions between the Two Groups

There were 2 cases of nausea and vomiting and 1 case of dizziness in the control group. In the observation group, there were 3 cases of dizziness and headache. There was no significant difference in the incidence of postpartum adverse reactions between the two groups (*χ*2 = 0.174 and *P* = 0.676). There were no serious adverse reactions such as mental symptoms and respiratory depression in the two groups of puerperae.

## 4. Discussion

Postpartum depression mainly refers to a depression that exists during the puerperium. During the onset of postpartum depression, persistent emotional depression is the main symptom and manifestation, accompanied by changes in thinking and behavior. According to the survey data, in my country, the incidence of postpartum depression is as high as 6.15% to 33.93% [5]. At the same time, clinical data show that the occurrence of postpartum depression on the one hand can have a large and small impact on the physical and mental health of puerperae. On the other hand, postpartum depression can threaten the baby's personality, cognitive ability, and behavioral training [6]. Therefore, it is of great significance to take active and effective preventive measures for the occurrence and development of depression after cesarean section.

The article "A Study on the Preventive Effect of Esketamine on Postpartum Depression (PPD) after Cesarean Section" was retracted in 2023. Reasons: unreliable results or conclusions; concerns about the data; concerns about the peer review; concerns about the citations.

In the current clinical work, although the antidepressant drugs taken can achieve a certain antidepressant effect, but antidepressant drugs have general flaws, mainly manifested in a delay of several weeks before it can take effect. In particular, some mothers who need to breastfeed have obvious rejection of most antidepressant drugs [7, 8]. Ketamine hydrochloride was first developed by Parke Davis in 1962 and belongs to a class of derivatives of phencyclidine (PCP). Ketamine hydrochloride is mainly used for anesthesia and has achieved good effects. Subsequently, after the acquisition of ketamine hydrochloride by Pfizer, a dextrorotatory split of ketamine (esketamine), was developed to exert a stronger and safer analgesic effect [9, 10], clinical data show that esketamine has stronger affinity and potency than ketamine hydrochloride. In addition, the pharmacokinetics of esketamine are controllable, and it can also achieve good results in the treatment of treatment-resistant depression [11, 12]. The mechanism of action of ketamine hydrochloride in the prevention and control of depression and its related symptoms lies in the inactivation of eukaryotic elongation factor-2 kinase through enhanced blocking of NMDA receptors. The inactivation of eukaryotic elongation factor-2 kinase reduces the level of eukaryotic elongation factor-2, avoids the increase of BDNF expression, and finally achieves the purpose of anti-depression. But whether ketamine hydrochloride can play an antidepressant effect after cesarean section is still worthy of research and analysis [13, 14]. Therefore, this study analyzed the preventive effect of esketamine on the occurrence of PPD after cesarean section. The results showed that the SBP, DBP, and HR of the observation group were higher than those of the control group at T4 and T5 time points. There was no significant difference in SBP, DBP, and HR at T3, T4, and T5 time in the observation group. Compared with T3, SBP, DBP, and HR were lower in control group T4 and T5, respectively. It can be seen that the application of esketamine can better ensure the stability of the patient's heart rate and blood pressure. And there is no increase in adverse reactions during the treatment period, ensuring the safety of the drug during the application period. When observing depressive symptoms, it can be seen that the EPDS score of the observation group was lower than that of the control group and the incidence of postpartum depression was higher at 3d and 42d postpartum. The results confirmed that esketamine has a strong antidepressant effect and effect and the depressive symptoms of some puerperae were relatively relieved, which was basically consistent with previous reports [15, 16]. At the same time, esketamine has a faster action speed and a relatively longer action time and has more comprehensive advantages. However, some experts believe that esketamine itself has a strong stimulating effect on the sympathetic nerve, which can easily lead to abnormally high blood pressure in mothers. Therefore, during the use of esketamine, it is necessary to comprehensively evaluate various basic indicators of cesarean section and select an appropriate dose to ensure better tolerance and safety for puerperae [17, 18].

The article "A Study on the Preventive Effect of Esketamine on Postpartum Depression (PPD) after Cesarean Section" was retracted in 2023. Reasons: unreliable results or conclusions; concerns about the data; concerns about the peer review; concerns about the citations.

In conclusion, the application of esketamine after cesarean section can effectively reduce depression-related scores and the risk of postpartum depression. And esketamine does not increase adverse reactions and has high safety. In the following clinical work, the sample size can be further expanded, the observation indicators can be increased, and the follow-up time can be extended, so as to better comprehensively evaluate the application effect of esketamine after cesarean section.

## Figures and Tables

**Table 1:** Comparison of general data between the two groups.

Groups	*N*	Age (year)	Body mass index kg/m^2^)	Gestational week (week)	Cesarean section implementation time (min)	Postoperative analgesic drug usage (ml)	Education level (below junior high school/high school/college and above)
Control group	69	29.21 ± 2.14	24.25 ± 1.21	39.10 ± 1.02	53.35 ± 10.25	110.39 ± 10.77	7/30/32
Research group	69	29.02 ± 2.33	24.30 ± 1.09	39.05 ± 0.99	53.10 ± 11.02	109.24 ± 12.31	10/32/27
t/*χ*^2^		0.490	0.255	0.292	0.138	0.584	1.012
p		0.619	0.799	0.771	0.891	0.560	0.601

**Table 2:** Comparison of changes in blood pressure and heart rate between the two groups.

Groups	*N*	Time point	SBP (mmHg)	DBP (mmHg)	HR (every time/min)
Control group	69	T1	108.44 ± 8.24	68.87 ± 9.23	86.10 ± 16.58
		T2	109.51 ± 9.87	66.20 ± 7.25	87.14 ± 14.20
		T3	111.54 ± 8.60	68.14 ± 8.36	87.65 ± 16.87
		T4	103.87 ± 12.54	62.54 ± 11.35	77.29 ± 11.20
		T5	105.54 ± 9.61	65.97 ± 11.66	80.03 ± 10.98
F			2.251	2.336	2.571
P			0.024	0.035	0.040
Research group	69	T1	112.02 ± 8.31	69.10 ± 10.21	87.56 ± 16.54
		T2	108.36 ± 9.64	67.22 ± 9.54	88.24 ± 15.60
		T3	112.02 ± 8.55	69.21 ± 8.30	89.36 ± 18.34
		T4	111.24 ± 12.98	71.39 ± 11.24	92.47 ± 11.87
		T5	108.77 ± 9.54	68.33 ± 10.77	90.54 ± 10.73
F			3.012	3.247	3.559
P			0.034	0.046	0.047

**Table 3:** Comparison of EPDS scores before and after cesarean section between the two groups (points).

Groups	*N*	Prenatal 1d	Postpartum 3d	Postpartum 42d
Control group	69	7.21 ± 4.24	8.66 ± 2.07	9.16 ± 2.01
Research group	69	7.18 ± 4.06	7.79 ± 2.14	8.43 ± 2.26
*t*		0.043	2.427	2.005
*P*		0.966	0.017	0.047

The article "A Study on the Preventive Effect of Esketamine on Postpartum Depression (PPD) after Cesarean Section" was retracted in 2023. Reasons: unreliable results or conclusions; concerns about the data; concerns about the peer review; concerns about the citations.

**Table 4:** Comparison of the incidence of depression after cesarean section between the two groups.

Groups	N	Prenatal 1d	Postpartum 3d	Postpartum 42d
Control group	69	6(9.09)	17(24.64)	15(21.74)
Research group	69	5(7.25)	7(10.14)	6(9.09)
*χ* ^2^		0.099	3.957	4.550
*P*		0.753	0.047	0.033

## Data Availability

Data to support the findings of this study is available on reasonable request from the corresponding author.
